This article has been retracted.

# Volleyball Sports Teaching Based on Augmented Reality and Wireless Communication Assistance

**DOI:** 10.1155/2022/9080602

**Published:** 2022-08-13

**Authors:** Wei Ding, Hao Li, Xi Wang

**Affiliations:** ^1^Department of Physical Education, Honam University, Gwangju Metropolitan City 62397, Republic of Korea; ^2^Department of Sports Welfare Education, Woosuk University, Jeonju 55338, North Jeolla, Republic of Korea; ^3^Basic Teaching Department of Qingdao University of Science and Technology, Weifang 261500, Shandong, China

## Abstract

The 21st century is the information age. The ever-changing information technology not only affects the development of the global economy, but also has an important impact on the field of education and personnel training. Under the influence of information technology, the way people acquire, impart, and evaluate knowledge has changed greatly. The educational concepts, models, and methods of the new era are fundamentally different from traditional education, which provides new opportunities and new challenges for the education and teaching work of contemporary teachers. This paper aims to discuss the application of augmented reality technology in volleyball teaching, and give an effective method for AR to be applied to volleyball teaching. In this paper, the existing AR teaching system has the problem of poor transmission rate and cannot cooperate with volleyball teaching well. Therefore, a wireless communication auxiliary algorithm based on intelligent reflective surface is proposed. And the current situation of volleyball teaching is investigated and analyzed. And in response to the survey results, 78% of the students supported teachers in applying AR technology to assist teaching in volleyball teaching classes. This fully shows that there is still a lot of application space for AR technology in current volleyball teaching.

## 1. Introduction

With the rapid development of modern education, information technology has become an indispensable part of the field of education and an important symbol of educational modernization. High school volleyball has the characteristics of comprehensiveness and regionality, abstract knowledge, and great difficulty in learning. The application of information technology to volleyball teaching has become the trend of the times. Based on reading a large number of related literatures, this paper clarifies the research topic and summarizes the background, significance, and research status of the application of augmented reality technology in high school volleyball teaching. Since the early domestic researches were mainly focused on children's education and higher education, factors such as the psychological laws of middle school students, the hardware facilities of ordinary middle schools, and the curriculum standards of middle schools were not well considered. Therefore, it is difficult to promote and popularize the results of early research in secondary education. Therefore, this paper is based on the teaching practice of high school volleyball, supported by constructivism theory, situational learning theory and audio-visual teaching theory, designed a research plan and carried out teaching experiments, and applied augmented reality technology to the teaching practice of high school volleyball.

Under the background of the times and the requirements of new curriculum standards, it is hoped that through this research, volleyball teachers can improve their ability to effectively use information-based teaching resources, especially the ability to effectively use AR technology. It also hopes to provide reference for volleyball teachers to transform teaching methods through AR technology, promote the transformation of volleyball teaching mode, cultivate students' information literacy, enhance students' volleyball thinking, change students' learning behavior, and improve students' volleyball practice ability.

The innovation of this paper is that: design teaching cases according to the teaching status and technology application status reflected by the survey data and carry out teaching experimental research on this basis. Combining teaching theory and teaching practice, this paper analyzes the effect of augmented reality technology in volleyball teaching from three aspects: volleyball test scores, student questionnaires, and teacher interviews. This paper points out the main factors that restrict the wide application of augmented reality technology in volleyball teaching, and provides real data and reference for front-line volleyball teachers to apply augmented reality technology to assist teaching. However, due to the small research scope and limited research time, the research conclusions of this paper also have certain limitations and one-sidedness. It is believed that with the rapid development of education modernization, the application of augmented reality technology in high school volleyball teaching will become more and more extensive and mature.

## 2. Related Work

As one of the three major balls, volleyball is widely loved. In particular, the spirit of the Chinese women's volleyball team has stimulated people's enthusiasm for volleyball, and there are many teaching and research on volleyball. The Batez study investigated the impact of a Teaching Play (TGfU) model implemented in physical education classes on volleyball skills and enjoyment of middle school students. The findings demonstrate the effectiveness of the short-term TGfU model (12 lessons) in improving volleyball skills in an educational setting. He also emphasized the importance of having fun in these classes compared to traditional physical education classes [1]. In order to help individuals deal with volleyball learning and training, Duan designed an online volleyball distance teaching system based on Augmented Reality (AR) technology [2]. Wang conducted a statistical empirical analysis on comprehensive strength and volleyball teaching evaluation based on regression model. The optimized traditional teaching evaluation system can improve the effectiveness of volleyball teaching evaluation, stimulate students' interest in learning volleyball, and provide necessary reference for volleyball teaching [3]. Wang and Liang studied the extraction method and teaching method of volleyball spiking trajectory based on wireless sensor network [4].

The research on augmented reality is also a current hot issue. AR is widely used, and there are many problems to be solved at the technical level, and there are many applications in teaching. Research by Paraskevaidis and Fokides presented the results of a pilot project using 360 videos to teach students basic volleyball skills [5]. Turkan et al. introduces a new structural analysis pedagogy that combines mobile augmented reality (AR) and interactive 3D visualization techniques [6]. Cabero-Almenara et al.'s research is part of the Spanish research project (I + D + I), which is part of augmented reality to facilitate training. Cabero-Almenara et al. aimed to study augmented reality for the Spanish project (I + D + I) to promote the design, production, and evaluation of augmented reality for university education. His results show that augmented reality is an emerging technology with broad training possibilities. However, it requires training and financial investment to guarantee its success in the classroom [7]. Research on AR technology in the field of education has the following characteristics: a late start, few achievements, and rapid progress. Since the early domestic researches were mainly focused on children's education and higher education, their research failed to take into account factors such as the psychological development of middle school students, the hardware facilities of ordinary middle schools, and the curriculum standards of middle schools. Therefore, the early research results are difficult to promote and popularize in middle schools, which makes the development and application of AR technology in the field of middle school education particularly lagging behind. Therefore, under the situation that AR technology is becoming more and more mature and the teaching effect is constantly being verified, it is necessary to transfer the application research of AR technology in education and teaching from the laboratory to the real middle school classroom, and from the colleges and universities to ordinary middle schools. Giving full play to the educational advantages of AR technology is exactly the research significance and purpose of this paper. However, it can be found that although there are many researches on volleyball teaching at present, most of them are limited to the use of technical means to improve the training level of athletes.

## 3. Augmented Reality and Volleyball Teaching

### 3.1. Application of Augmented Reality in Teaching

AR technology is a technology with interactive functions that superimposes virtual information into the real environment with the support of related equipment, so that the virtual information and the real environment are presented synchronously in the same time and space. It is related to VR technology but it is different, as shown in Figure 1.

AR technology is built on the basis of reality, and it is still the real world at all. Its simple schematic diagram is shown in Figure 2.

As shown in Figure 2, AR technology mainly has the following characteristics. (1) Interactivity: AR technology can superimpose virtual information and real environment into the same space. With the support of corresponding interactive hardware devices and AR software systems, users can realize real-time interactive activities with the superimposed virtual-real synchronized environment. The interactivity of AR technology can be realized in any real environment and is not limited by time and space. The interactive characteristics of AR technology have greatly changed the user experience, making users change from noninteractive communication with the screen to interactive activities with the help of AR devices. Users can integrate with the real environment after superimposing virtual information through interactive activities and can also directly interact with the augmented reality environment through the use of body movements, language commands and other methods, which greatly improves the user's technical experience. (2) Immersion: AR technology can place users in a real environment superimposed with virtual information. This unique immersion feature can help students immerse themselves in the learning situation created by AR technology, so as to help students achieve the purpose of active inquiry, active learning, and active thinking. In the learning situation created by AR technology, students change from passively receiving knowledge to actively acquiring knowledge. With the continuous progress and innovation of AR technology, the learning situations created by AR technology are becoming more and more realistic, and the depth of immersion is continuously enhanced. The deeply immersive learning environment is very helpful for students to understand knowledge, just like the audience's viewing experience. The deeper the immersion in the plot, the easier it is for the audience to understand the development of the plot. Likewise, the more immersed a student is in the learning situation created by AR, the easier it will be to comprehend the knowledge. (3) Connectivity between virtual and real: AR technology can realize real-time synchronization of virtual information and real environment, and also realize the three-dimensional presentation of virtual information and real environment in the same time and space. The ever-changing AR technology can well realize the connection between virtual information and the real environment, which greatly reduces the sense of violation of the virtual-real connection in the AR experience process [8, 9]. For students, AR technology can superimpose the complex and incomprehensible abstract knowledge with large time and space scales with the real environment of the real world in a virtual presentation way, so as to realize the connection between virtual information and the real environment. It can help students' experience and observe complex and abstract knowledge in various learning situations created by AR technology. This feature of AR technology is of great help to students' learning.

With the development of modern educational technology, the application of Augmented Reality (AR) technology has also begun to penetrate into the field of education. The American New Media Alliance has twice listed AR technology as a new technology that will have an important impact on modern education in the Horizon Report. AR technology has accumulated a lot of experience worthy of reference in various learning modes such as game learning and interactive learning, and successfully and effectively integrated digital teaching resources with the real world. And it produces educational products such as popular AR books, AR educational software, and AR educational games. It can be seen that the rise of AR technology has laid a good foundation for its application in the field of education. AR technology can superimpose abstract volleyball knowledge, especially the larger space-time scale, into the real environment, and students can observe, experience, and understand the knowledge immersive in the augmented reality world. It creates an advantage condition that other technologies cannot match for volleyball teaching. Facing the rapid rise of AR technology, volleyball teachers should take a positive attitude to meet the opportunities and challenges that AR technology brings to volleyball education. The application of AR in teaching is shown in Figure 3 [10, 11].

### 3.2. Feasibility of AR Applied to Volleyball Teaching

#### 3.2.1. Augmented Reality Application Equipment is Simple

With the rapid development of AR technology, there are more and more devices supporting AR technology, including professional equipment such as AR glasses, AR helmet, and AR projector, as well as smart mobile devices such as mobile phones and tablet computers that realize augmented reality functions through camera functions. Among the above equipments, due to the high price of professional equipment, they have not been widely used. Therefore, AR technology based on smart mobile devices such as mobile phones and tablet computers has become the most commonly used and mainstream augmented reality method due to its easily acceptable price and good augmented reality effects. It can be seen that it is not difficult to apply AR technology to education and teaching. Only a smartphone or tablet with a camera function and AR application software can effectively complete classroom teaching, so that students can get AR learning experience in the classroom, as shown in Figure 4.

#### 3.2.2. Abundant Educational Products of Augmented Reality

Since the most common and mainstream augmented reality method is realized through mobile devices such as mobile phones and tablet computers, there are many AR education products developed and designed based on mobile devices. Thanks to the development and popularization of smart mobile devices and network communication technology, coupled with the increasingly mature AR technology, teachers of various disciplines can now choose AR products suitable for their classrooms from the rich and diverse AR education software to assist teaching. In terms of middle school volleyball teaching, more mature products have been developed: “Understanding Junior High School Volleyball” for junior high school volleyball and “AR Middle School Globe” for high school volleyball. In addition, teachers can also try to independently develop and create simple AR materials according to teaching needs and teaching material content [12]. Currently, the design platforms available for teachers to develop AR resources include ARToolKit, BuildAR, Sky Eye AR, and Vision + AR. Blippbuilder has also opened an AR development platform that does not require programming for nonprofessional users. The rich and diverse AR software and development platforms provide a strong technical guarantee for the application of AR technology in education and teaching.

#### 3.2.3. Augmented Reality Technology Has a Wide Range of Applications

AR technology can transform abstract content into concrete images due to its good interactivity, immersion, and virtual-real connectivity. The application of AR technology is of great significance to overcoming the above difficult knowledge and cultivating students' spatial imagination. It can be seen that the application scope of AR technology in volleyball teaching is very broad, and the application significance is very significant [13].

### 3.3. Wireless Communication Auxiliary System

Although the global deployment of fifth-generation mobile communications (5G) has just started, industry and academia have begun to look to the post-5G future, such as sixth-generation mobile communications (6G), which are designed to meet higher requirements than 5G. 6G requires higher throughput, higher energy efficiency, wider connectivity, and higher reliability and lower latency than 5G. However, the existing 5G technologies are mainly aimed at the three major application scenarios of enhanced mobile broadband (eMBB), ultra-reliable and low-latency communication (URLLC), and massive machine communication (mMTC), which may not fully meet the requirements of 6G [14, 15]. The main reasons are as follows: First, the existing 5G technology achieves an increase in network coverage and capacity by deploying more active nodes to form an ultra-dense network. Deploying more active nodes also leads to higher energy consumption, higher deployment, feedback and maintenance costs, and more severe and complex network interference problems. Second, by installing more antennas on active nodes such as base stations, access points, and relays, performance gains are obtained by forming massive multiple-input multiple-output (MIMO). However, deploying large-scale antennas will greatly increase the power consumption, hardware cost, and signal processing complexity of the system. In addition, by mining new spectrum resources, such as resources in higher frequency bands such as millimeter wave (mmWave) or even terahertz (THz), to solve the problem of scarce spectrum resources. However, high-frequency communication has serious path loss, and in order to compensate for the path loss, it is usually necessary to deploy more active nodes or configure more antennas [16, 17].

Intelligent Reflector (IRS) can realize intelligent control of wireless propagation environment, provides an important technical solution to solve the above problems, and has become a key candidate technology in 6G. A typical IRS is a plane composed of a large number of low-cost, almost passive reflectors. Each reflector can independently control changes in the amplitude and/or phase of the incident signal. By densely deploying IRS in a wireless network and intelligently coordinating its reflections, the wireless channel between transmitter and receiver can be flexibly controlled to achieve the desired signal propagation environment. Thereby, it provides a new method to fundamentally solve the problem of wireless channel fading and interference, and it is possible to realize a huge leap in the throughput and reliability of wireless communication network.

Figure 5 shows a typical architecture of IRS [18]. The outermost panel is composed of a large number of almost passive reflective elements to achieve direct interaction with the incident signal. The main function of the middle panel is to avoid leakage of signal energy. The inner panel is the control circuit, which adjusts the reflection coefficient of the reflection element through the IRS controller. In practice, a programmable gate array (FPGA) can be used as the IRS controller. In addition, the IRS controller can communicate and coordinate with other network components (such as BS) through a separate feedback link, enabling low-rate information exchange. Figure 5 also shows an example of the structure of reflectors, each controlled by a switching diode [19]. By controlling the bias voltage through the DC feeder, the switching diode can be switched between “on” and “off” states, resulting in a phase difference of *π*. By setting the corresponding bias voltage through the IRS controller, the phase shift of each reflector can be adjusted independently. In order to control the amplitude of the reflection coefficient, a variable resistance load can be used in the design of the reflection element, and the amplitude and phase shift of the inverse element can be changed by changing the resistance value. Therefore, the above circuit needs to be effectively integrated.

To address the above two problems, this chapter proposes a novel location-based multi-IRS-assisted multiuser system framework. The proposed location information-based design framework has the following three advantages over existing design frameworks, which require complete CSI and consume a large amount of pilot overhead. First, location data can be easily collected via GPS, significantly reducing pilot overhead. Second, unlike instant CSI, location information changes slowly, so it does not need to be constantly updated. In addition, since only a limited amount of location data needs to be transmitted between the base station and the IRS, only a small-capacity feedback link is required, thereby reducing the installation cost of the IRS. In the following introduction, the abbreviations and symbols involved are shown in Tables 1 and 2.

As shown in Figure 6, this chapter considers a multi-IRS-assisted multiuser system in which a BS with N antennas communicates with *K* single-antenna users, each assisted by an IRS with *M* reflectors. The BS is connected to the IRS via a low-capacity hardware link to exchange information (such as CSI and phase shift information) with each other.

Using Rice fading to model the channels from BS to IRS and from IRS to users:

(1) $$\begin{array}{c} G_{B2I,m}=\sqrt{\frac{\alpha_{B2I,m}v_{B2I,m}}{v_{B2I,m}+1}}{\bar{G}}_{B2I,m}+\sqrt{\frac{\alpha_{B2I,m}}{v_{B2I,m}+1}}{\tilde{G}}_{B2I,m}. \end{array}$$

Among them,

(2) $$\begin{array}{c} {\tilde{G}}_{B2I,m}\in C^{M\times N}. \end{array}$$

Formula (2) represents the NLoS component, each element of which obeys a complex Gaussian distribution *CN*(0,1), *α*_*B*2*I*,*m*_ represents large-scale fading, *v*_*B*2*I*,*m*_ represents the Rice factor, and the LoS component ${\bar{G}}_{B2I,m}$ is expressed as

(3) $$\begin{array}{c} {\bar{G}}_{B2I,m}=b\left(\theta_{y-B2Ia,m}\right)a^{T}\left(\theta_{y-B2I,m}\right). \end{array}$$

The effective departure angle can be expressed as

(4) $$\begin{array}{c} \theta_{y-B2I,m}=-\frac{2\pi d_{BS}}{\lambda }\cos\theta_{B2I,m}\sin\theta_{B2I,m}, \end{array}$$

*d*_*BS*_ represents the distance between the adjacent antennas of the BS. Similarly,

(5) $$\begin{array}{c} b\left(\theta_{y-B2Ia,m}\right)\in C^{M\times 1}. \end{array}$$

The effective departure angle is expressed as

(6) $$\begin{array}{c} \theta_{y-B2Ia,m}=\frac{2\pi d_{\text{IRS}}}{\lambda }\cos\theta_{B2Ia,m}\sin\theta_{B2Ia,m}. \end{array}$$

*d*_*IRS*_ represents the distance between adjacent reflectors, cos  *θ*_*B*2*Ia*,*m*_sin  *θ*_*B*2*Ia*,*m*_ are the elevation and azimuth angles of the *m*th IRS, respectively. Also, assume:

(7) $$\begin{array}{c} d_{\text{IRS}}=d_{BS}\\ =\frac{\lambda }{2}. \end{array}$$

The *n*-th element of the array response vector *a*(*ϑ*) and the *l*-th element of *b*(*ϑ*) are given by the following two equations, respectively,

(8) $$\begin{array}{c} a_{n}=e^{j\pi \left(n-1\right)\theta },\;n=1,\ldots ,N,\\ b_{l}=e^{j\pi \left(l-1\right)\theta },\;l=1,\ldots ,M. \end{array}$$

Similarly, the channel from the *m*th IRS to the *k*th user is expressed as

(9) $$\begin{array}{c} g_{12U,mk}^{T}=\sqrt{\frac{\alpha_{12U,mk},v_{12U,mk}}{v_{12U,mk}+1}}{\bar{g}}_{12U,mk}^{T}+\sqrt{\frac{\alpha_{12U,mk}}{v_{12U,mk}+1}}{\tilde{g}}_{12U,mk}^{T}. \end{array}$$

Among them, the LoS component is

(10) $$\begin{array}{c} {\bar{g}}_{12U,mk}^{T}\in C^{1\times M}. \end{array}$$

It can be expressed as:

(11) $$\begin{array}{c} {\bar{g}}_{12U,mk}^{T}=b^{T}\left(\theta_{y-12U,mk}\right). \end{array}$$

The BS sends a signal:

(12) $$\begin{array}{c} X=\sum_{i=1}^{K}w_{i}s_{i}. \end{array}$$

Among them,

(13) $$\begin{array}{c} w_{i}\in C^{N\times 1}. \end{array}$$

Formula (13) represents the base station transmit beam, satisfying:

(14) $$\begin{array}{c} E\left\{{\left|s_{i}\right|}^{2}\right\}=1. \end{array}$$

The signal received by the *k*th user can be expressed as

(15) $$\begin{array}{c} y_{k}=\sum_{m=1}^{K}\sum_{i=1}^{K}g_{12U,mk}^{T}\Theta_{m}G_{B2I,m}w_{i}s_{i}+n_{k}. \end{array}$$

Among them, *n*_*k*_ ∈ *CN*(0, *σ*_0_^2^) represents AWGN, and the phase shift matrix of the *m*th IRS is

(16) $$\begin{array}{c} \Theta_{m}=\text{diag}\left(\xi_{m}\right)\in C^{M\times M}. \end{array}$$

Among them,

(17) $$\begin{array}{c} \xi_{m}={\left[e^{j\Theta_{m},1},\ldots ,e^{j\Theta_{m},n},\ldots ,e^{j\Theta_{m},M}\right]}^{T}\in C^{M\times 1}. \end{array}$$

Formula (17) represents the IRS passive beam.

### 3.4. Algorithm Simulation Results

Figure 7 shows the system and rate for different Rice factors. It can be seen that the numerical results are in complete agreement with the analytical results, thus verifying the correctness of the analytical expressions. Due to the combined effect of interuser interference and leakage power, the sum rate saturates at high SNR. Also, as the uncertainty of the user's location increases, the sum rate decreases significantly.

Figure 8 depicts the performance of the proposed beamforming technique compared to the best power control scheme in this paper. All users are assumed to have the same desired rate. The joint optimization technique of the study was used as a benchmark, and many IRSs were considered to be one giant distributed IRS. It can be seen that the proposed scheme significantly outperforms the baseline scheme when the desired rate is not very high. With a small rate limit, the required transmit power is not high, so the system is likely to be noise limited. In noise-constrained environments, systems based on maximum ratio combining (MRC) are close to ideal. This is then combined with an optimal power control algorithm to improve results. However, when the rate limit is tightened, the necessary transmit power goes up and the system is hindered by interference. Due to significant interference, the performance of the planned MRC scheme gradually degrades and falls short of the baseline scheme. Also, if the desired rate exceeds a certain threshold, the optimization problem may not be solved. The reason is that beamforming techniques were not developed with interference suppression in mind, which can only be partially corrected by using power control and deploying IRS locations in a logical manner. In other words, deploying a large number of IRS in all directions, increasing the distance between them, and assigning each user to the IRS closest to them. On the other hand, the baseline system uses perfect CSI and combinatorial optimization methods to iteratively solve two SDP subproblems to optimize active and passive beams. The results show that the baseline method can better tolerate interuser interference.

## 4. Investigation on the Application of AR Technology in Volleyball Teaching

### 4.1. Experimental Method

Questionnaire survey method: A questionnaire about volleyball learning and the application of AR technology in high school volleyball teaching was distributed in the No. 6 Middle School in K City, to investigate the basic situation of students' volleyball learning and the application status of AR technology in high school volleyball teaching.

Interview method: According to the interview outline, the volleyball teachers in K city were interviewed, and from the perspective of teachers, the current situation of teachers using information technology to assist volleyball teaching and the application status of AR technology in high school volleyball teaching were investigated.

There are 15 questions in the questionnaire, all of which are multiple-choice questions. The main survey contents are volleyball learning interest (questions 1-2); learning difficulty (questions 3–5); classroom atmosphere (questions 6-7); teaching methods (questions 8–11); teaching effect (question 12); students' understanding of AR technology (question 13); the application of AR technology (question 14); students' attitude towards the application of AR technology in the classroom (question 15).

There are 6 questions in the interview outline. The main content of the interview is the current situation of high school volleyball teaching, including teachers' teaching methods, teaching methods, understanding of AR technology, application of AR technology, and attitude towards the application of AR technology in teaching.

### 4.2. Survey Results

The questionnaire survey is to randomly select 100 students in K city to distribute paper questionnaires. A total of 100 questionnaires were distributed in this survey, and 98 were recovered, of which 95 were valid questionnaires. With the help of SPSS software and EXCEL software to carry out statistics and analysis on the results of the questionnaire, the analysis results are as follows.

#### 4.2.1. Survey on Students' Interest in Volleyball Learning

Questions 1-2 mainly focus on volleyball learning interest. The survey results show that among the students surveyed, 28% of the students are not very interested in volleyball, and 52% of the students are more interested in volleyball, 12% of students have no interest in volleyball, while only 8% are very interested in volleyball. Among the factors that affect students' interest in volleyball lessons, the volleyball classroom atmosphere is the most influential factor with 44% of paired interest in volleyball learning. Secondly, the teaching method of teachers accounted for 30%, the content of teachers' teaching accounted for 20%, and some other factors such as: the degree of love for volleyball teachers, the amount of homework, and the difficulty of homework. The above data shows that most students are highly interested in volleyball learning, and only a small number of students are not interested in volleyball. Compared with the teaching content, students are more concerned about the classroom atmosphere and teachers' teaching methods. In addition, students' evaluation of teachers and after-school homework also constitute factors that affect students' interest in volleyball learning. The details are shown in Tables 3 and 4.

#### 4.2.2. Survey on Volleyball Classroom Atmosphere

Questions 6-7 mainly focus on the volleyball classroom atmosphere. The survey results show that 46% of the students ideally have a more active volleyball classroom atmosphere, 41% of the students hope that the volleyball classroom is very active, 9% of the students like the classroom atmosphere of occasional communication, and only 4% of the students want the volleyball classroom to be very quiet. In fact, only 18% of the students expected the volleyball classroom atmosphere to meet their expectations. 58% of the students believed that the volleyball classroom atmosphere was sometimes what they expected, and 24% of the students believed that the current volleyball classroom atmosphere was not what they expected at all. The above data shows that students prefer a relatively active classroom atmosphere to a very active or very quiet classroom atmosphere. The actual volleyball classroom atmosphere is relatively dull and quiet, and students' expectations can only be met occasionally, which also provides a good opportunity for the application of AR technology in teaching, as shown in Tables 5 and 6.

#### 4.2.3. Survey on Students' Understanding of AR Technology

Question 13 mainly surveys students' understanding of AR technology. The survey results show that 54% of students have never used AR technology in their life, 40% of students have used AR technology occasionally, and only 6% of students often use AR technology. The above data shows that there are more students who are infrequently exposed to AR technology than those who are often exposed to AR technology, and most students lack understanding of AR technology. Only a very small number of students often use AR technology and mainly understand the technology through AR games, and have not used AR technology in their studies. It can be seen that although AR technology has developed very maturely and is widely used in various aspects, AR technology is still a relatively unfamiliar technology to students in K City. On the one hand, the application of new technology can help teachers solve volleyball teaching problems and improve teaching efficiency. On the other hand, it is also helpful to increase students' interest in volleyball learning and mobilize students' enthusiasm and initiative in learning, which is also one of the necessary reasons for AR technology to be applied to volleyball teaching.

Question 14 mainly investigates the application of AR technology in volleyball teaching. According to the survey results, 94% of the students chose that teachers have never used AR technology in volleyball lessons, 6% of students chose teachers to occasionally use AR technology in volleyball lessons, and no students chose teachers to use AR technology frequently. The above data shows that the application of AR technology in the current volleyball classroom is very small, and only some teachers occasionally try to use it. It can be seen that the application status of AR technology in the current volleyball teaching is not ideal, and the specific reasons will be further understood through interviews with teachers.

Question 15 mainly surveys students' attitudes towards the application of AR technology in the classroom. The survey results show that 78% of students support teachers' application of AR technology in volleyball classes to assist teaching, 13% of students think it doesn't matter, and 9% of students do not support teachers' application of AR technology in class. The above data shows that most students have a positive attitude towards the application of AR technology, which creates a good atmosphere for the application of AR technology, as shown in Figure 9.

### 4.3. Suggestions on AR Application in Volleyball Teaching

In order to ensure the smooth application of AR technology in volleyball teaching, it is necessary to improve technical support first, such as multimedia resources and the introduction of advanced AR technology. First of all, it is necessary to introduce foreign advanced hardware equipment and development platforms, so that students have a sense of “reality” in the electronic environment. Therefore, it is necessary to introduce foreign advanced technology to improve the equipment platform for information collection, processing, and display. Secondly, the design should be “usefulness, usability, and emotionality.” The application of AR technology in volleyball teaching should design a concise interface and operation process. So, it can make the combination of virtual and reality, and the combination of AR technology and traditional classroom teaching bring vivid interactive emotional experience. From the perspective of visual elements, the use of augmented reality technology to break through the visual expression of traditional classroom teaching, and replace it with a dynamic, virtual and realistic visual image to express the language of information. In terms of auditory elements, real and natural sounds are applied in teaching with the help of augmented reality technology, so as to endow volleyball teaching with vitality and lasting vitality.

## 5. Conclusion

In China, AR teaching research is in its infancy. Although various disciplines have achieved different degrees of research results in related fields, the current research in various fields is still immature, and the majority of educators still need to continue to explore and practice to provide useful guidance for the application of AR technology in the field of education. This paper firstly investigates the current status of volleyball teaching and the application status of AR technology in volleyball teaching. Firstly, this paper investigates the current situation of volleyball teaching and the application of AR technology in volleyball teaching, and designs teaching cases according to the investigation results, and then carry out teaching experimental research through the method of quasiexperimental research, and evaluate the effect of AR technology applied to high school volleyball teaching in multiple ways, aiming to provide reference and reference for the application of AR technology in high school volleyball teaching.

## Figures and Tables

**Figure 1:** AR and VR.

**Figure 2:** AR principle.

**Figure 3:** AR applied to teaching.

**Figure 4:** AR applied to volleyball.

**Figure 5:** Typical architecture of the IRS.

**Figure 6:** Multi-IRS-assisted multiuser system.

**Figure 7:** System and rate at different settings.

**Figure 8:** Performance of the beamforming scheme.

**Figure 9:** Students' understanding of AR.

**Table 1:** Abbreviation comparison table.

Abbreviate	English full name
AWGN	Additive white Gaussian noise
BS	Base station
CSI	Base station
IRS	Intelligent reflecting surface
ULA	Uniform linear array
LOS	Line-of-sight

**Table 2:** Symbol comparison table.

Symbol	Meaning
*a*	Vector *a*
*A*	Matrix *A*
*E*{}	Mathematical expectation
*θ*	The complexity
diag (*A*)	Diagonal operations
*C* ^*M*×*k*^	*M* × *N* matrices over the complex field
CN (*µ*, Σ)	Complex Gaussian distribution
*N*(*µ*, Σ)	Gaussian distribution

**Table 3:** Students' interest in volleyball lessons.

Attributes	Percentage (%)
A. Very interested	8
B. More interested	52
C. Not very interested	28
D. Have no interest	12

**Table 4:** Factors affecting students' interest in volleyball lessons.

Attributes	Percentage (%)
A. The way teachers teach	30
B. Teachers teach content	20
C. Volleyball classroom activity level	44
D. Other	6

**Table 5:** Students' expectations for the classroom atmosphere of volleyball teaching.

Attributes	Percentage (%)
A. Very active	41
B. Is more active	46
C. Occasional communication	9
D. No communication	4

**Table 6:** Does the volleyball classroom atmosphere meet student expectations?

Attributes	Percentage (%)
A. Very satisfied	18
B. Relatively satisfied	58
C. Not satisfied	24

## Data Availability

The data that support the findings of this study are available from the corresponding author upon reasonable request.
